The article "Da Vinci Robot-Assisted Video Image Processing under Artificial Intelligence Vision Processing Technology" was published in 2022. Journal: Comput Math Methods Med.

# Da Vinci Robot-Assisted Video Image Processing under Artificial Intelligence Vision Processing Technology

**DOI:** 10.1155/2022/2752444

**Published:** 2022-04-30

**Authors:** Qiangli Cheng, Yajun Dong

**Affiliations:** ^1^Department of Medical Equipment, The First Affiliated Hospital of University of South China, Hengyang, 421001 Hunan, China; ^2^Department of Medical Equipment, The Second Affiliated Hospital of University of South China, Hengyang, 421001 Hunan, China

## Abstract

This research was aimed to explore the application value of intelligent algorithm-based digital images in Da Vinci robot-assisted treatment of patients with gastric cancer surgery. 154 patients were included as the research objects, with 89 cases in the control group underwent laparoscopic surgery, and 65 cases in the experimental group underwent robotic surgery. According to the propensity score, the patients in two groups were pair matched (1: 1), of which 104 cases (52 cases in each group) were successfully matched. The general data of patients, the changes in the images before and after the algorithm processing, the intraoperative and postoperative conditions, the pathological examination results, and the follow-up information were observed after matching. Compared with the original images, the images processed by the thread image edge detection algorithm had the significantly improved clarity, as well as highly reduced artifacts and noises. The sensitivity, specificity, and accuracy of image-assisted diagnosis were improved remarkably, showing the differences of statistical significance (*P* < 0.05). The total time of surgery, intraoperative bleeding, CRP (1d and 3d after surgery), and postoperative total abdominal drainage showed the significant differences as well (*P* < 0.05). The surgeries of patients in both groups met R0 resection (no tumor infiltration within 1 mm of the surgical margin), but there was a significant difference in the number of lymph node dissections (*P* < 0.05). The overall survival rates of patients in the experimental group and the control group were 83.0% and 76.1%, respectively, 2 years after surgery, with no significant difference (*P* > 0.05). The thread image edge detection algorithm produced a better processing effect on the images, which greatly improved the diagnostic sensitivity, specificity, and accuracy. Compared with endoscopic surgery, robotic surgery has better postoperative recovery, safety and reliability, and obvious advantages of minimally invasive surgery.

## 1. Introduction

In the medical industry, the minimally invasive surgeries are increasing. Compared with traditional open surgery, it does not require a large incision for the operation. Therefore, it has the advantages of smaller incision that can reduce the harm to the patients, shorten hospitalization time to promote the recovery of patients, and reduce the possibility of bacterial infection by reducing blood transfusion. Meanwhile, it also has an exclusive advantage on medical cosmetology [1, 2]. In recent years, intelligent health care has gradually come into the life; with the booming medical robot market, the development of artificial intelligence technology has brought new opportunities to the robot industry [3]. Da Vinci robot, as the bellwether in surgical robots, almost monopolizes the market as the robotic surgical system in the highest level is presented. Da Vinci robot includes 3 core techniques: freely swinging arms, three-dimensional high-definition video image technology, and human-computer interaction design of the main control console. It can simulate the various operation modes of the human arm with 7 degrees of freedom [4, 5]. When the operation is deep in the body, it will be more accurate than that operated manually due to its compact and flexible characteristics. It can also eliminate the situation of hands tremble occurs during manual surgery, which expands the accuracy and safety of surgery [6].

The article "Da Vinci Robot-Assisted Video Image Processing under Artificial Intelligence Vision Processing Technology" was published in 2022. Journal: Comput Math Methods Med.

With the third technological revolution, computer technology and image processing technology have been improved. The performances of optical instruments have also been greatly improved, promoting machine vision technology with rapid development [7]. The technical core of the thread image edge detection algorithm is the digital image processing technology, which is inseparable from the computer technology. Its main characteristics include complete processing techniques, considerable starting and running speed, excellent image processing effect, and the matched functional response to software changes [8]. Meanwhile, for the continuous upgrades of optical components and integrated circuits, the continuous advancement of digital scientific theories, and the continuous expansion of national production and defense reserves, this technology receives unprecedented attention to make many algorithms have the strong robustness and better processing effect [9].

So far, the digital image processing technology has been widely used in important fields such as industrial detection, medical imaging, remote sensing satellites, and national defense [10]. It is highly dependent on image measurement technology, which is on the basis of optical equipment and related theoretical knowledge. The image measurement technology combines computer, optoelectronics, laser, and other technologies for comprehensive applications, with the advantages of high accuracy and fast speed. Its essence is to select a suitable image processing algorithm for the target image processing, so that the relevant image area is free from noises; then, the image of the measurement object is segmented and extracted; and corresponding algorithms are used to measure parameters [11, 12]. For improving the accuracy and efficiency of image measurement, it is necessary to analyze the characteristics of each object to be measured in detail and select the corresponding optimal method.

The article "Da Vinci Robot-Assisted Video Image Processing under Artificial Intelligence Vision Processing Technology" was published in 2022. Journal: Comput Math Methods Med.

Gastric cancer is a common malignant tumor of the digestive system, which mostly occurs on the side of the lesser curvature of the gastric antrum. In recent years, the incidence and mortality of gastric cancer have been increasing, which shows a trend of the patients getting younger and younger [13]. Nowadays, the treatment of gastric cancer is still based on radical resection, combined with a multidisciplinary diagnosis and treatment model. As the main development direction of gastrointestinal surgery, minimally invasive surgery has an irreplaceable position [14]. In 2002, the first global report was made on the Da Vinci robotic surgery system for gastric cancer radical resection [15]. In this research, 154 gastric cancer patients were included as the research objects. 89 patients who received radical distal gastrectomy with laparoscopy were in the control group, while the other 65 patients who underwent radical distal gastrectomy with the Da Vinci robotic surgery system were in the experimental group. A thread image edge detection algorithm was proposed for image enhancement processing, to analyze the application value of the intelligent algorithm-based digital images deeply in Da Vinci robot-assisted treatment of patients with gastric cancer surgery.

## 2. Research Objects

### 2.1. General Data of Patients

The clinicopathological data of 154 patients with gastric cancer were collected, and the patients were admitted to the hospital from January 2019 to March 2021. There were 95 males and 59 females, with the median age of 54 years old, and the age ranged from 36 to 80 years old. 89 patients who underwent radical resection using laparoscopy were taken as the control group, and 65 patients who underwent radical resection using the Da Vinci robotic surgery system were included in the experimental group. According to the inclusion criteria, patients diagnosed with gastric cancer by gastroscopy were included, and it was determined they would have the radical distal gastrectomy. Preoperative-enhanced computerized tomography (CT) examination of the chest and abdomen showed no distant metastases to the liver, lung, or other organs, as well as no invasion to pancreas. They had not undergone any surgery or severe inflammation in the chest and abdomen in the medical history, and they offered the complete clinicopathological data. With the exclusion criteria, patients with multiple primary tumors, distant metastasis, or gastric remnant cancer were excluded. Patients with contraindications to laparoscopic surgery were also excluded, such as patients cannot tolerate general anesthesia and patients with blood coagulation disorders and portal hypertension. Those patients with incomplete clinical data were not included as well. All the cases included and their families consented to this study, and they signed the informed consent forms. This study has been approved by the medical ethics committee of hospital.

The article "Da Vinci Robot-Assisted Video Image Processing under Artificial Intelligence Vision Processing Technology" was published in 2022. Journal: Comput Math Methods Med.

### 2.2. Surgical Methods

The willingness of the patients and their families were taken into consideration, so they underwent the traditional laparoscopic surgery or Da Vinci robotic surgery as they selected. According to the research of Chen et al. (2020) [16], all patients underwent distal subtotal gastrectomy and D2 lymph node dissection. The laparoscopic radical surgeries of gastric cancer were operated based on the *Laparoscopic Gastric Cancer Surgery Guidelines (2016 Edition)* formulated by the Laparoscopic Surgery Professional Committee of Chinese Medical Association (CMA). Da Vinci robotic surgery system for the radical surgeries of gastric cancer was run on the *Expert Consensus of Robotic Gastric Cancer Surgery (2015 Edition)* of the Robotics Committee of the Chinese Research Hospital Association (CRHA). Through the auxiliary small incision in the upper abdomen, the tumor tissues were removed, and the digestive tract was reconstructed during the surgery. The digestive tract reconstruction adopted the Billroth I and Billroth II methods, in which the digestive tract was anastomosed with a 25-mm tubular round stapler. The digital images before and during the surgery were processed by the thread image edge detection algorithm.

### 2.3. Thread Image Edge Detection Algorithm

Firstly, for the pixel-level edge detection, differential operator was fundamental and important. It was very sensitive to noise and included Marr algorithm, Krish algorithm, Roberts algorithm, Canny algorithm, and gradient algorithm. The Canny algorithm had the good reliability and practicability, and could extract image information accurately, which mainly involved in the following aspects.

After the binarized image was input, the Gaussian-Laplace second-order differential filter was used to obtain the following

(1) $$\begin{array}{c} g\left(z\right)=\frac{1}{\sigma^{3}\sqrt{2\pi }}e^{-\frac{z_{2}}{2\sigma_{2}}}\left(\frac{z^{2}}{\sigma^{2}}-1\right). \end{array}$$

After smoothing process of the image, the following equation is obtained.

(2) $$\begin{array}{c} R\left[k,l\right]=G\left(k,l;\sigma \right)*K\left(k,l\right), \end{array}$$

where *K*(*k*, *l*) stands for the original image, *G*(*k*, *l*; *σ*) is the Fourier transform of the two-dimensional function extended by Equation (1), *σ* is the variance of the Gaussian function, and *R*[*k*, *l*] represents the two arrays *P*[*k*, *l*] and *Q*[*k*, *l*] of *z* and *o* partial derivatives, which were obtained using 2 × 2 finite difference of first-order partial derivative. The two arrays were expressed as

(3) $$\begin{array}{c} P\left[k,l\right]\approx \frac{\left(R\left[k,l+1\right]-R\left[k,l\right]+R\left[k+1,l+1\right]-R\left[k+1,l\right]\right)}{2}, \end{array}$$

(4) $$\begin{array}{c} Q\left[k,l\right]\approx \frac{\left(R\left[k,l\right]-R\left[k+1,l\right]+R\left[k,l+1\right]-R\left[k+1,l+1\right]\right)}{2}. \end{array}$$

At this time, the gradient magnitude and direction could be worked out by

(5) $$\begin{array}{c} A\left[k,l\right]=\sqrt{P{\left[k,l\right]}^{2}+Q{\left[k,l\right]}^{2}}, \end{array}$$

(6) $$\begin{array}{c} \theta \left[k,l\right]=\arctan\left(\frac{Q\left[k,l\right]}{P\left[k,l\right]}\right). \end{array}$$

Then, the edge width was adjusted to be a single pixel through the nonmaximum suppression method. This process was called nonmaximum suppression.

The article "Da Vinci Robot-Assisted Video Image Processing under Artificial Intelligence Vision Processing Technology" was published in 2022. Journal: Comput Math Methods Med.

For the improvement of the positioning accuracy, the double-threshold detection method was used to filter out false edges. There were two thresholds in this method, namely, a high threshold and a low threshold. If the high threshold was less than the pixel gradient value, the pixel was marked as an edge. If the gradient value was less than the low threshold, it was marked as a nonedge point. If the gradient value was between the two thresholds, it was judged whether the pixel was connected to the obtained edge. If it was, it was marked as an edge, and finally, the pixel-level edge was obtained.

In this study, the following equation is used to test the performance of Canny algorithm, and *Q* refers to the quality coefficient of the processed image.

(7) $$\begin{array}{c} Q=\left(\frac{1}{\max\left\{a,b\right\}}\right)\overset{b}{\underset{k=1}{\sum }}\left[\frac{1}{\left(1+\alpha \times d^{2}\left(k\right)\right)}\right], \end{array}$$

where *a* is the number of theoretical edges, *b* is the actual number of edges extracted by the Canny algorithm, *d*(*k*) represents the distance between the Image-th edge and the corresponding actual edge, and *α* is the constant of proportionality, with a value of 0.1 generally.

The article "Da Vinci Robot-Assisted Video Image Processing under Artificial Intelligence Vision Processing Technology" was published in 2022. Journal: Comput Math Methods Med.

After test, the image quality coefficient *Q* = 0.9543, which was close to 1, indicating that the edge extracted by the Canny algorithm was close to the actual edge.

The interpolation-based subpixel positioning technology was the most commonly used subpixel edge positioning method currently, with a good calculation efficiency. Before this technology was put into use, the pixel-level edge had to be extracted via the Canny algorithm. Meanwhile, the original grayscale image *f*(*k*, *l*) and original gradient image *S*(*k*, *l*) were computed by the Sobel algorithm, as shown in

(8) $$\begin{array}{c} S\left(k,l\right)=\left|f\left(k-1,l-1\right)-f\left(k+1,l+1\right)\right|+\left|f\left(k-1,l+1\right)-f\left(k+1,l-1\right)\right|, \end{array}$$

(9) $$\begin{array}{c} S\left(k,l\right)=\left|\begin{array}{c} f\left(k+1,l+1\right)+2f\left(k,l+1\right)+f\left(k-1,l+1\right)\\ -f\left(k-1,l-1\right)-2f\left(k,l-1\right)-f\left(k+1,l-1\right) \end{array}\right|+\left|\begin{array}{c} f\left(k-1,l-1\right)+2f\left(k-1,l\right)+f\left(k-1,l+1\right)\\ -f\left(k+1,l+1\right)-2f\left(k+1,l\right)-f\left(k+1,l-1\right) \end{array}\right|. \end{array}$$

If the point (*a*, *b*) was confirmed as an edge point, then three points *S*(*a* − 1, *b*), *S*(*a*, *b*), and *S*(*a* + 1, *b*) were taken along the *Z* direction of the gradient image *S*(*k*, *l*). Their gradient magnitudes were regarded as the function values. *m* − 1, *m*, and *m* + 1 were taken as the interpolation base points and put into the quadratic polynomial *ψ*(*z*) with *dψ*(*z*)/*dx* = 0. Similarly, three points *S*(*a*, *b* − 1), *S*(*a*, *b*), and *S*(*a*, *b* + 1) were taken in the *O* direction, and the same calculation process was performed to obtain the subpixel edge coordinates (*Z*_*p*_, *O*_*p*_). The calculation is as follows:

(10) $$\begin{array}{c} \psi \left(z\right)=\overset{2}{\underset{k=0}{\sum }}\overset{2}{\underset{k=0,l\neq k}{\prod }}\frac{z-z_{k}}{z_{k}-z_{l}}o_{k}, \end{array}$$

where *z*_*k*_ and *o*_*k*_ represent the interpolation base point and the function value, respectively. Then, the equations are worked out as follows:

(11) $$\begin{array}{c} \left\{\begin{array}{c} Z_{p}=a+\frac{S\left(a-1,b\right)-S\left(a+1,b\right)}{2\left[S\left(a-1,b\right)-2S\left(a,b\right)+S\left(a+1,b\right)\right]}\\ O_{p}=b+\frac{S\left(a,b-1\right)-S\left(a,b+1\right)}{2\left[S\left(a,b-1\right)-2S\left(a,b\right)+S\left(a,b+1\right)\right]} \end{array}\right., \end{array}$$

(12) $$\begin{array}{c} S\left(a,b\right)>S\left(a-1,b\right),S\left(a,b\right)>S\left(a+1,b\right), \end{array}$$

(13) $$\begin{array}{c} S\left(a,b\right)>S\left(a,b-1\right),S\left(a,b\right)>S\left(a,b+1\right). \end{array}$$

The article "Da Vinci Robot-Assisted Video Image Processing under Artificial Intelligence Vision Processing Technology" was published in 2022. Journal: Comput Math Methods Med.

### 2.4. Observation Indicators

For the comparison of patients' general data, the patients in two groups were pair matched (1 : 1) according to the propensity score. The comparison was made after the matching, in the age, gender, body mass index (BMI), preoperative C-reactive protein (CRP), carcino-embryonic antigen (CEA), tumor diameter, and tumor-node-metastasis (TNM) staging of patients. For the image processing results of thread image edge detection algorithm, the sensitivity, specificity, and accuracy of the images before and after processing were observed [17]. The intraoperative and postoperative situations of patients in the two groups were also compared after the propensity score-based matching. The comparisons were in terms of the total time of surgery, the dissociation time in vivo, intraoperative bleeding, CRP (1d and 3d after surgery), postoperative total abdominal drainage, drainage tube removal time after surgery, the time of the first gas exhaustion by anus after surgery, the incidence of postoperative complications, and the hospitalization time. After the matching, patients' pathological examination results were compared as well. It was studied whether patients in the two groups met R0 resection, which required no tumor infiltration within 1 mm of the surgical margin. The number of lymph node dissections was also analyzed via the examination. After the patients were matched, the number of medical staff in the follow-up, the duration of follow-up, the incidence of complications during the follow-up, and the survival condition of patients were compared between two groups. Through outpatient or telephone follow-ups, the incidence of serious complications and the survival condition of patients after discharge were known. The overall survival time referred to the time from the day of surgery to the last follow-up or the death of a patient.

### 2.5. Statistical Analysis

All the data in this study were analyzed through SPSS 19.0. The nearest neighbor matching method in Empower Stats software was used for the 1 : 1 pair matching of patients in the two groups based on the propensity scores. The mean ± standard deviation was used to represent the measurement data in the normal distribution, and the *t* test was used for the comparisons between two groups. In the skew distribution, *M* (range) represented the measurement data, and Mann–Whitney *U* test was used to compare the data between two groups. The absolute value, the *χ*^2^ test, and the Mann–Whitney *U* test were applied for the enumeration data, the corresponding comparisons between two groups, and the comparison of the ranked data between two groups, respectively. The survival rate was calculated through the Kaplan-Meier method, and the log-rank test was used for survival analysis. *P* < 0.05 indicated that the difference was statistically significant.

The article "Da Vinci Robot-Assisted Video Image Processing under Artificial Intelligence Vision Processing Technology" was published in 2022. Journal: Comput Math Methods Med.

## 3. Results

### 3.1. Comparison of General Data of Patients

After matching, the age, gender, BMI, CRP, CEA, tumor diameter, and TNM staging of patients in the two groups were compared. The comparisons are shown in Figures 1, 2, and 3 in details.

From Figures 1, 2, and 3, for patients in this study, there is no statistically significant difference in their age, gender, BMI, preoperative CRP, CEA, tumor diameter, and TNM staging between the experimental group and the control group (*P* > 0.05).

### 3.2. Image Processing of Thread Image Edge Detection Algorithm

Laparoscopic images of the patients are processed by the thread image edge detection algorithm in this study, and the results are shown in Figures 4 and 5. After the images were processed by the thread image edge detection algorithm, the image definition was significantly improved. The sensitivity, specificity, and accuracy of the images were also greatly improved, and the differences were all significant statistically (*P* < 0.05).

### 3.3. Intraoperative and Postoperative Conditions of Patients

After the patients in the two groups were matched, the intraoperative and postoperative conditions of patients are compared, as shown in Figures 6, 7, and 8 in detail. The items compared included the total time of surgery, dissociation time in vivo, blood loss during surgery, CRP (1d and 3d after surgery), postoperative total abdominal drainage, drainage tube removal time postoperatively, the time of the first gas exhaustion by anus after surgery, the incidence of postoperative complications, and hospitalization time.

From Figures 6, 7, and 8, it is suggested that there were significant differences in the total time of surgery, intraoperative bleeding, CRP (1d and 3d after surgery), and the postoperative total abdominal drainage of patients between the two groups, and the differences were statistically significant (*P* < 0.05). However, the differences were not obvious (*P* > 0.05) in the dissociation time in vivo, drainage tube removal time, the time of the first gas exhaustion by anus, the incidence of postoperative complications, and hospitalization time of patients between the two groups.

### 3.4. Pathological Examination of Patients

After the propensity score-based matching, the patients in the two groups were examined to discover whether the R0 resection was achieved on them, with the standard for no tumor infiltration within 1 mm of the gastric and duodenal surgical margin. The number of lymph node dissections was also observed. More details are shown in Table 1.

The article "Da Vinci Robot-Assisted Video Image Processing under Artificial Intelligence Vision Processing Technology" was published in 2022. Journal: Comput Math Methods Med.

As shown in Table 1, the standard of R0 resection is reached for patients in both groups. But there was a statistically significant difference in the number of lymph node dissections (*P* < 0.05) between the two groups.

### 3.5. Follow-Up Information

All the 104 matched patients were followed up after surgery for 5-38 months. All the patients had no serious complications, such as obstruction of afferent/efferent loop and dumping syndrome, within 12 weeks after the surgery. The postoperative overall survival rates of patients in the two groups are shown in Figure 9. As shown in Figure 9, the overall survival rates of patients in the experimental group and the control group are 83.0% and 76.1%, respectively, and there is no significant difference between the groups (*P* >0.05).

## 4. Discussion

Da Vinci robot consists of three parts: the surgeon console, the bedside robotic arm system, and the imaging system. Since it was approved for clinical use by the Food and Drug Administration (FDA) in 2000, there are increasing reports of it on radical resection of gastric cancer [18]. In this study, propensity score matching reduced the confounding effect and balanced differences between the two groups effectively, having a wide range of applications globally. The important indicators for evaluating the feasibility and safety of a surgical method are the total time of the surgery and the intraoperative bleeding. It was reported that compared with traditional laparoscopic surgery, the robotic surgery system could give a longer total time of the radical resection of gastric cancer, but the volume of intraoperative bleeding would be reduced using a robot [19].

Research of Cui et al. (2020) [20] showed that there was a significant difference in the total time of surgery between the robotic surgery system and the traditional laparoscopic surgery, and the time was longer than that in this study. The reason was that the ranges of gastrectomy in the two researches were different. Relevant studies have shown no statistically significant difference in the actual time of gastrectomy between robotic surgery system and traditional laparoscopic surgery [21]. For this reason, the time of surgery was further studied, and no significant difference was found in the dissociation time in vivo of patients between the two groups (*P* > 0.05). However, the total time of surgery for the patients in two groups was significantly different. Compared with those in the control group, patients in the experimental group had less intraoperative bleeding and more lymph node dissections (*P* < 0.05), which was similar to the results obtained by Pan et al. This was due to the mechanical advantages of the robotic surgery system. While the difficulty of the surgery was reduced, it could clean the lymph nodes in the pylorus, the upper edge of the pancreas, and so on more accurately and carefully; thereby, the damage to the microvessels was reduced. It was observed that the Da Vinci robotic surgery system had obvious advantages in lymph node dissection and surgical operations of complex parts.

The article "Da Vinci Robot-Assisted Video Image Processing under Artificial Intelligence Vision Processing Technology" was published in 2022. Journal: Comput Math Methods Med.

Another key factor in evaluating the quality of surgery is the postoperative recovery [22]. This study showed that, compared with the results in the control group, patients in the experimental group had less total abdominal drainage after surgery, but the difference in drainage tube removal time was not statistically significant. Perhaps this was because the Da Vinci robot could make the perigastric mesentery keep smooth during the radical resection of gastric cancer, which made the mesenteric space separation more precise. It was beneficial to the off-bed activity of patients as the abdominal drainage tube was pulled out as earlier as possible under safe conditions after surgery, which promoted the recovery of respiratory and digestive functions and reduced the incidence of complications as well. Relevant reports indicated that there was no significant difference in the incidence of complications after the radical resection of gastric cancer between using the robotic system and laparoscope [23], which was consistent with the results of this study. The CRP of patients in the experimental group (1d and 3d after surgery) was relatively less than those in the control group. Thus, the Da Vinci robotic surgery system had a smaller impact on physical indicators of patients in the radical resection of distal gastric cancer, showing the significant minimally invasive advantages. After the matching under propensity scores, there was no significant difference in the overall survival rate of patients in the 2 years after surgery between the experimental group and the control group (*P* > 0.05). The existing researches pointed out no statistically significant difference in the long-term efficacies of advanced gastric cancer with laparoscopic surgery and traditional open surgery [24]. It was concluded that the Da Vinci robotic surgery system was the same as laparoscopic surgery in terms of radical resection of distal gastric cancer. It was safe and reliable, with a similar short-term survival effect.

## 5. Conclusion

In this study, the thread image edge detection algorithm was utilized to process the digital images, and the application effect of the Da Vinci robotic surgery system in the treatment of radical resection of distal gastric cancer was studied. The sensitivity, specificity, and accuracy of the image processed by the algorithm were improved significantly, indicating that the image display under the algorithm was better. The postoperative recovery of patients treated by the robot was better than that after laparoscopic surgery, which suggested the robotic surgery system was safe and reliable with distinct minimally invasive advantages. However, due to the relatively small sample size and short follow-up time, the long-term efficacy needed to be verified by more clinical trials. Therefore, more patients will be included in the follow-up work, and a multicenter and controlled intervention research will be conducted. In conclusion, the results of this work provided a reference for the application of intelligent algorithms combined with Da Vinci robot in clinical surgery.

The article "Da Vinci Robot-Assisted Video Image Processing under Artificial Intelligence Vision Processing Technology" was published in 2022. Journal: Comput Math Methods Med.

## Figures and Tables

**Figure 1:** Comparison of the patients' age and gender in the two groups.

**Figure 2:** BMI, preoperative CRP, tumor diameter, and CEA of patients in two groups.

**Figure 3:** Comparison of TNM staging of patients in the two groups.

**Figure 4:** Images before and after algorithm processing which (a) indicated the images before processing and (b) showed the images after processing. The arrow in each image pointed to the lesion.

**Figure 5:** Sensitivity, specificity, and accuracy of the images before and after processed using the thread image edge detection algorithm. ∗# meant *P* < 0.05, which suggested the differences were statistically significant.

**Figure 6:** Total time of surgery, dissociation time in vivo, and intraoperative bleeding of patients between the two groups. ∗# meant *P* < 0.05 with statistically significant differences.

**Figure 7:** CRP 1d and 3d after surgery and the time of the first gas exhaustion by anus of patients in the two groups: (a) displayed the CRP level, while (b) was of the time of the first gas exhaustion by anus. ∗# indicated *P* < 0.05, as the differences were statistically significant.

**Figure 8:** Total abdominal drainage, drainage tube removal time, hospitalization time, and the incidence of complications of patients between the two groups after surgery. ∗# showed *P* < 0.05, for the difference was statistically significant.

**Figure 9:** Overall survival rates of patients in the two groups after surgery.

**Table 1:** Pathological examination results of patients in the two groups.

Groups	R0 resection	Number of lymph node dissections
The experimental group	Met the standard	23 ± 3
The control group	Met the standard	21 ± 3

## Data Availability

The data used to support the findings of this study are available from the corresponding author upon request.
